This article has been retracted.

# Repurposing food molecules as a potential BACE1 inhibitor for Alzheimer’s disease

**DOI:** 10.3389/fnagi.2022.878276

**Published:** 2022-08-22

**Authors:** Nobendu Mukerjee, Anubhab Das, Rahul D. Jawarkar, Swastika Maitra, Padmashree Das, Melvin A. Castrosanto, Soumyadip Paul, Abdul Samad, Magdi E. A. Zaki, Sami A. Al-Hussain, Vijay H. Masand, Mohammad Mehedi Hasan, Syed Nasir Abbas Bukhari, Asma Perveen, Badrah S. Alghamdi, Athanasios Alexiou, Mohammad Amjad Kamal, Abhijit Dey, Sumira Malik, Ravindra L. Bakal, Adel Mohammad Abuzenadah, Arabinda Ghosh, Ghulam Md Ashraf

**Affiliations:** ^1^Department of Microbiology, Ramakrishna Mission Vivekananda Centenary College, Khardaha, India; ^2^Department of Health Sciences, Novel Global Community Educational Foundation, Hebersham, NSW, Australia; ^3^Institute of Health Sciences, Presidency University, Kolkata, India; ^4^Department of Medicinal Chemistry, Dr. Rajendra Gode Institute of Pharmacy, Amravati, India; ^5^Department of Microbiology, Adamas University, Kolkata, India; ^6^Central Silk Board, Guwahati, India; ^7^Institute of Chemistry, University of the Philippines Los Baños, Los Baños, Philippines; ^8^Department of Pharmaceutical Chemistry, Faculty of Pharmacy, Tishk International University, Erbil, Iraq; ^9^Department of Chemistry, Faculty of Science, Imam Mohammad Ibn Saud Islamic University, Riyadh, Saudi Arabia; ^10^Department of Chemistry, Vidya Bharati Mahavidyalaya, Amravati, India; ^11^Department of Biochemistry and Molecular Biology, Faculty of Life Sciences, Mawlana Bhashani Science and Technology University, Tangail, Bangladesh; ^12^Department of Pharmaceutical Chemistry, College of Pharmacy, Jouf University, Sakaka, Saudi Arabia; ^13^Glocal School of Life Sciences, Glocal University, Saharanpur, India; ^14^Department of Physiology, Faculty of Medicine, King Abdulaziz University, Jeddah, Saudi Arabia; ^15^Pre-Clinical Research Unit, King Fahd Medical Research Center, King Abdulaziz University, Jeddah, Saudi Arabia; ^16^The Neuroscience Research Unit, Faculty of Medicine, King Abdulaziz University, Jeddah, Saudi Arabia; ^17^Department of Science and Engineering, Novel Global Community Educational Foundation, Hebersham, NSW, Australia; ^18^AFNP Med, Vienna, Austria; ^19^Institutes for Systems Genetics, Frontiers Science Center for Disease-Related Molecular Network, West China Hospital, Sichuan University, Chengdu, China; ^20^King Fahd Medical Research Center, King Abdulaziz University, Jeddah, Saudi Arabia; ^21^Department of Pharmacy, Faculty of Allied Health Sciences, Daffodil International University, Dhaka, Bangladesh; ^22^Enzymoics, Novel Global Community Educational Foundation, Hebersham, NSW, Australia; ^23^Department of Life Sciences, Presidency University, Kolkata, India; ^24^Amity Institute of Biotechnology, Amity University, Jharkhand, Ranchi, India; ^25^Department of Medical Laboratory Sciences, Faculty of Applied Medical Sciences, King Abdulaziz University, Jeddah, Saudi Arabia; ^26^Microbiology Division, Department of Botany, Gauhati University, Guwahati, India

**Keywords:** beta-site APP cleaving enzyme 1, BACE1, Alzheimer’s disease, glioblastoma, QSAR, molecular docking, MD simulations, golden lotus banana

## Abstract

Alzheimer’s disease (AD) is a severe neurodegenerative disorder of the brain that manifests as dementia, disorientation, difficulty in speech, and progressive cognitive and behavioral impairment. The emerging therapeutic approach to AD management is the inhibition of β-site APP cleaving enzyme-1 (BACE1), known to be one of the two aspartyl proteases that cleave β-amyloid precursor protein (APP). Studies confirmed the association of high BACE1 activity with the proficiency in the formation of β-amyloid-containing neurotic plaques, the characteristics of AD. Only a few FDA-approved BACE1 inhibitors are available in the market, but their adverse off-target effects limit their usage. In this paper, we have used both ligand-based and target-based approaches for drug design. The QSAR study entails creating a multivariate GA-MLR (Genetic Algorithm-Multilinear Regression) model using 552 molecules with acceptable statistical performance (*R*^2^ = 0.82, *Q*^2^_*loo*_ = 0.81). According to the QSAR study, the activity has a strong link with various atoms such as aromatic carbons and ring Sulfur, acceptor atoms, sp2-hybridized oxygen, etc. Following that, a database of 26,467 food compounds was primarily used for QSAR-based virtual screening accompanied by the application of the Lipinski rule of five; the elimination of duplicates, salts, and metal derivatives resulted in a truncated dataset of 8,453 molecules. The molecular descriptor was calculated and a well-validated 6-parametric version of the QSAR model was used to predict the bioactivity of the 8,453 food compounds. Following this, the food compounds whose predicted activity (pKi) was observed above 7.0 M were further docked into the BACE1 receptor which gave rise to the Identification of 4-(3,4-Dihydroxyphenyl)-2-hydroxy-1H-phenalen-1-one (PubChem I.D: 4468; Food I.D: FDB017657) as a hit molecule (Binding Affinity = −8.9 kcal/mol, pKi = 7.97 nM, Ki = 10.715 M). Furthermore, molecular dynamics simulation for 150 ns and molecular mechanics generalized born and surface area (MMGBSA) study aided in identifying structural motifs involved in interactions with the BACE1 enzyme. Molecular docking and QSAR yielded complementary and congruent results. The validated analyses can be used to improve a drug/lead candidate’s inhibitory efficacy against the BACE1. Thus, our approach is expected to widen the field of study of repurposing nutraceuticals into neuroprotective as well as anti-cancer and anti-viral therapeutic interventions.

## Graphical Abstract

Food molecules as a potential BACE1 inhibitor against Alzheimer’s disease.

## Introduction

Alzheimer’s disease (AD) is a devastating mental illness, which leads to an irreversible, progressive brain disorder that slowly destroys memory skills and learning abilities (De Strooper and Karran, 2016). Though the disease progression and risk factors of AD are not completely understood, a large number of evidence suggest the formation of amyloid-beta (Aβ) is central to the pathophysiology of AD (Vassar et al., 1999). AD progression stages vary from mild to severe in middle-aged people to older persons detected with cognitive tests (Hall et al., 2019). During the preclinical stage of AD, patients seem to be symptom-free, but neurodegenerative changes occur in the brain. Abnormal accumulation of Aβ-containing plaques and hyperphosphorylated tau throughout the brain causes healthy neurons to exhibit loss of synaptic connections, ion-channel dysfunctions, and severe deterioration in neuronal health. This ultimately leads to neuronal cell death and cognitive decline in elderly persons (Musi et al., 2018; Sebastián-Serrano et al., 2018). This progressive accumulation of Aβ is caused by imbalances in the levels of Aβ production, aggregation, and clearance (Murphy and LeVine, 2010; Jabir et al., 2021). Moreover, alterations in synaptic plasticity and integral neuronal circuitries severely hamper neurogenesis.

The Special Report examines MCI, including Alzheimer’s, from the perspectives of consumers and primary care providers. AD affects 6.5 million Americans who are 65 years old or older. By 2060, this figure may increase to 13.8 million unless medical advances prevent, slow down, or cure AD. A total of 121,499 AD deaths were reported on official death certificates in 2019. According to one COVID-19 report, AD is the sixth most common cause of death in the United States in 2019 and will move up to the seventh most common cause in 2020 and 2021. Among Americans 65 and older, AD is the seventh most common cause of death. Between 2000 and 2019, mortality from HIV, heart disease, and stroke all dropped, whereas AD deaths rose by 145 percent. In 2021, 16 billion hours of care were supplied by over 11 million family members and other unpaid caregivers. These statistics demonstrate a decrease in carers and an increase in the amount of care that each caregiver who is still working gives. $271,6 billion was spent on unpaid dementia care in 2021. Family caregivers now have a higher risk of emotional discomfort as well as poorer mental and physical health due to COVID-19. Caregivers of dementia are also impacted by COVID-19. To safeguard their own health and the health of their families, several caregivers have resigned. However, there is a need for more dementia carers. Medicaid payments are more than 22 times greater than Medicare payments, and payments to beneficiaries 65 and older with AD or other dementias are approximately three times more than payments to beneficiaries without these illnesses. Hospice, long-term care, and healthcare for dementia patients will cost $321 billion in 2022. A poll by the Alzheimer’s Association indicates MCI obstacles. The study revealed low MCI knowledge, a lack of desire to seek medical attention for symptoms, and challenges with MCI diagnosis. According to survey findings, clinical trial participation should be increased together with MCI awareness and diagnosis, particularly in impoverished communities (Alzheimer’s Association, 2012).

Aβ is a neurotoxic aggregate produced by the consecutive proteolysis of β-amyloid precursor protein (APP) by two aspartyl proteases, beta-site APP cleaving enzyme, Beta-Secretase (BACE1), and finally by γ secretase (Sinha et al., 1999; Vassar et al., 1999; Yan et al., 1999; Cui et al., 2011; Zhang et al., 2011). BACE1 is a novel target, a type 1 transmembrane aspartic protease, related to the pepsin and retroviral aspartic protease families (Moussa-Pacha et al., 2020), having 501 amino acids and is predominantly expressed in the human brain (Zacchetti et al., 2007; Hassan et al., 2018).

As there is a strong association between Aβ accumulation and AD, the primary therapeutic strategy for the treatment of AD targets lowering the concentration of Aβ. One such strategy that has come up in recent findings involves inhibiting the enzymes that generate Aβ in the first place. BACE1 antisense oligonucleotide treatment to APP overexpressing cells is reportedly responsible for a decreased production of β-secretase cleaved APP fragments. Recent studies suggest that the levels of BACE1 protein and their activity were raised to approximately double in patients with AD where BACE1 might initiate or enhance AD pathogenesis. Several studies proved that BACE1 is a vital drug target and active site of the enzyme (Sinha et al., 1999; Vassar et al., 1999; Dingwall, 2001; Fukumoto et al., 2002; Yang et al., 2003; Li and Südhof, 2004). It is covered by a flexible antiparallel β-hairpin, called a flap (Hussain et al., 2000). It is elucidated that the flap can control substrate access to the receptor site and set the substrate into the perfect orientation for the catalytic process (Lin et al., 2000). Hence, the inhibition of proteases such as BACE1 may represent modifying treatment for AD by controlling the production of Aβ (Tresadern et al., 2011; Arif et al., 2020). Therefore, BACE1 inhibitors may be used to treat AD.

Natural compounds have been investigated for many years for their ability to target a range of *trans-*acetyl peptidases in the search for new medications with fewer side effects due to their high biocompatibility. Apart from their benefits, the majority of natural compounds have a variety of disadvantages, including a high molecular weight, low stability, and in many cases, insufficient solubility. These difficulties can be resolved by using computer-assisted research to generate more effective and selective inhibitors. They are less harmful and more readily absorbed into the body than manufactured drugs. Computational techniques enable the modeling and screening of such compounds in a cost-effective and informative manner from a vast library of choices. The binding sites for various bioactive substances in BACE1 protein were predicted, and their interactions were explored utilizing the Food database and molecular docking. *Musella lasiocarpa’*s bioactive component, 4-(3,4-Dihydroxyphenyl)-2-hydroxy-1H-phenalen-1-one, is found to be the potential inhibitor of BACE1. *M. lasiocarpa*, also known as Chinese Dwarf Banana, is the only species in the genus Musella, which belongs to the family of Musaceae. Some novel compounds have also been isolated from this plant, which showed remarkable *in vitro* anticancer activities and some degree of antimicrobial activity (Bo et al., 2000; Dong et al., 2011).

These results demonstrate the potential of the *M. lasiocarpa* as a source of novel drugs, nutraceuticals, and functional foods. The result from this study will inspire the perspective of natural compounds and computer-aided drug discovery and, in the long run, significantly reduce the time required to research and build new lead compounds with specified biological activity and structural variety.

## Methodology

### QSAR modeling

Organization for economic corporation and development guidelines and a standard protocol recommended by different researchers, which involved sequential execution of (1) data collection and its curation, (2) structure generation and calculation of molecular descriptors, (3) objective feature selection (OFS), (4) splitting the dataset into training and external validation sets, and (5) subjective feature selection involving building a regression model and validation of the developed model, has been followed to build a widely applicable QSAR model for the BACE1 inhibitory activity. This also ensures thorough validation and successful application of the model.

#### Selection of data set

The data set of BACE1 inhibitory activity used for building, training, and validating the QSAR model in the present work was downloaded from the Chembl database (accessed on 22nd December 2021)^1^, which is a free and publicly accessible database. Initially, the data set comprised of 552 molecules (Davies et al., 2015). Then, as a part of data curation, entries with ambiguous Ki values, duplicates, salts, metal-based inhibitors, etc., were omitted. The final data set comprises structurally diverse 371 molecules with remarkable variation in structural scaffolds, which were tested experimentally for potency in terms of Ki (nM). A collection of 371 molecules with various structural configurations with mentioned enzyme inhibitory concentration (Ki) was decided on for the existing work (O’Boyle et al., 2011; Tosco et al., 2011; Fujita and Winkler, 2016). The Ki values ranging from 0.47 to 1,400 nM have been transformed to pKi (pKi = – logKi) earlier than real QSAR evaluation for ease of dealing with the data. Five least and five most active molecules are depicted in Figure 1 to illustrate the version in bio-activity with chemical features. The SMILES strings with mentioned Ki and pKi values for all of the molecules are depicted inside Supplementary Table 1 with the Supplementary material.

**FIGURE 1:** Schematic representation of the inhibition of Aβ plaque formation by FDB017657.

#### Molecular structure drawing and optimization

Drawing the 2D structures of all 371 and converting them to their corresponding 3D structures was done using ChemSketch 12 Freeware and Open Babel 2.4, (O’Boyle et al., 2011) both free and open-source software, respectively.^2^ After that, the MMFF94 force field available in TINKER (default setting) and Open3DAlign is used for optimization and molecular alignment, respectively.

#### Molecular descriptor calculation and objective feature selection

PyDescriptor has over 30,000 molecular descriptors for each molecule (Masand and Rastija, 2017). Molecular descriptors with near constant values (>95%) and resonance (|R|) > 0.95 were eliminated using OFS in QSARINS v2.2.4 (Gramatica et al., 2013, 2014). This work removed duplicate molecular descriptors and prevented collisions of multicollinearity and hypothetical variables in the Genetic Algorithm multiple linear regression (GA-MLR) model. Only 3,281 molecular descriptors were found in the reduced pool of molecular descriptors generated after OFS processing.

#### Subjective feature selection, QSAR model development, and validation

A reduced set of molecular descriptors consisting of 1D to 3D descriptors, molecular properties and charge descriptors, etc., covers a fairly complete descriptor space. A statistically robust genetic algorithm (GA) based on multiple linear regression (MLR) was deployed to run the QSAR model using the subjective feature selection (SFS) task in QSARINS v2.2.4. Models derived according to the organization for economic corporation and development (OECD) principles have been subjected to rigorous internal and external statistical validation, scrambling, and range analysis. The QSAR deployment process goes through the following steps:

To generate a QSAR model from the split data set, a random split operation is performed in QSARINS v2.2.4 to split the given data set into 80% training set (297 molecules) and 20% predictions (74 molecules set). A total of 297 molecules in the training set were used to develop the QSAR model, and external validation was performed on 74 molecules in the prediction set (Gramatica et al., 2013).

The GA-MLR-based QSAR model was built with the default setting QSARINS v2.2.4. Subjective feature selection was performed by setting Q^2^_LOO_ as a fitness feature. The Q^2^_LOO_ score increased significantly to six variables but then increased slightly. Therefore, to avoid overfitting the model, SFS was limited to a set of seven descriptors. This helped to get a simple and informative QSAR model (see Supplementary Table 2 in Supplementary Information) for additional information on the six selected molecular descriptors present in the QSAR).

A good QSAR model which has been properly validated using various methods such as cross-validation, external validation, Y-randomization, and applicability domain (Williams plot) is useful for future utilization in virtual screening, molecular optimization, and decision making, etc. The following statistical parameters and their recommended threshold values are routinely used to validate a model (Bellacasa et al., 2013; Roskoski, 2013; Fujita and Winkler, 2016; Gramatica, 2020): R^2^_tr_ ≥ 0.6, Q^2^_loo_ ≥ 0.5, Q^2^_LMO_ ≥ 0.6, *R*^2^ > Q^2^, R^2^_ex_ ≥ 0.6, RMSE_tr_ < RMSE_cv_, ΔK ≥ 0.05, CCC ≥ 0.80, Q^2^-_Fn_ ≥ 0.60, r^2^_m_ ≥ 0.5, (1-r^2^/r_o_^2^) < 0.1, 0.9 ≤ k ≤ 1.1 or (1-r^2^/r_o_^2^) < 0.1, 0.9 ≤ k’ ≤ 1.1,(r_o_^2^- r’_o_^2^|) < 0.3, RMSE_ex_, MAE_ex_, R^2^_ex_, Q^2*F*1^, Q^2^_F2_, Q^2^_F3_, and low R^2^_Yscr_, RMSE and MAE. The formulae for calculating these statistical parameters are available in Supplementary Table 3 in the Supplementary material. In addition, the Williams plot was plotted to evaluate the applicability domain of the QSAR model.

### QSAR-based virtual screening

A database of 26,467 food compounds was downloaded from FooDB (accessed December 28, 2021)^3^, primarily for QSAR-based virtual screening (VS) accompanied through the utility of Lipinski rule of five; the elimination of duplicates, salts, and metal derivatives resulted in a truncated dataset of 8,453 molecules. Therefore, the 8,453-food molecule was mainly used for VS-based QSAR. Prior to the calculation of the molecular descriptor, the 3D molecular system was organized within the same Method as a modeling set. Next, the molecular descriptor was calculated and a well-validated 6-parametric version of the QSAR model was used to predict the bioactivity of the new compound (Gramatica, 2013; Neves et al., 2018; Zaki et al., 2021; Jawarkar et al., 2022; Mukerjee et al., 2022). (The calculated molecular descriptors along with the predicted pKi and Ki values with smiles strings are given in Supplementary Table 4 in the Supplementary material).

### Virtual screening of natural compounds using molecular docking

The structure-based virtual screening of the compounds was performed using AutoDock vina Version 1.1.2 (Trott and Olson, 2010). Binding sites of BACE1 for screening were predicted using DoGSiteScorer (Volkamer et al., 2012) and information about the binding site of the native ligand. The size of the grid box was set to be 96 × 52 × 56 Å for BACE1, centered around the identified binding site. The compounds with the best binding affinity (kcal/mol) corroborating ligand-based screening in the QSAR analysis were selected for the studies.

### Preparation of protein and ligand molecule

The target of interest BACE1 (PDB I.D: 2ZHV) crystallographic structure was discovered in the Protein Data Bank’s structural database, and a molecular editor with an open-source license was used to import the structure (Discovery studio visualizer 4.0)^4^ (Figure 2). To get the structure optimized, the UCSF Chimera utilized the steepest descent to find 1,000 steps, followed by the conjugate gradient of energy minimization approach to optimize the structure of 4-(3,4-dihydroxyphenyl)-2-hydroxy-1H-phenalen-1-one (PubChem I.D: 4468; Food I.D: FDB017657) was acquired from Food Database after screening and QSAR. This dataset was imported into the DS visualizer and saved as PDB files.

**FIGURE 2:** Variations in activity and chemical structure in the present dataset of BACE1 inhibitors.

The FOOD database was used to obtain the library of ligands by screening the metabolites of *M. lasiocarpa* (Bonvino et al., 2018). The smiles notation and the three-dimensional structures of the selected ligands were downloaded in SDF format from the PubChem database (Kim et al., 2019), and further ligand structure files were converted to PDB format using Open Babel software (O’Boyle et al., 2011). The energy minimization of the ligands was performed in UCSF Chimera software (Pettersen et al., 2004) using the Amber ff 14 sb force field. The receptor used in the study is receptor tyrosine kinase; RCSB Protein Data Bank (PDB) (Berman et al., 2000) was used to download receptors BACE1 with PDB I.D: 2ZHV, Resolution: 1.85 Å. The protein structure was prepared by removing ligand, water molecules, and metal ions. Polar hydrogens were added, and non-polar hydrogens were merged. Finally, Kollman charges were added to the protein molecule before converting to PDBQT format by AutoDock Tools (v.1.5.6) of the MGL software package (Forli et al., 2016).

### Molecular docking for validation of docking score

The best hits from the QSAR modeling and virtual screening were re-docked against BACE1 (PDB I.D: 2ZHV). Protein and ligand preparations were done using AutoDock Tools (v.1.5.6) (Forli et al., 2016). Gasteiger charges were added to the ligand molecules prior converting to the PDBQT format. Online server DoGSiteScorer and the information about the binding site residues of native ligand were used to construct the grid box. The grid box of dimensions 96 × 52 × 56 Å for BACE1 with 0.375 Å grid spacing was constructed using auto grid 4.2. Semi-flexible docking was done keeping the receptor molecule rigid and ligands flexible. Molecular docking was done via AutoDock 4.2 (Morris et al., 2009) using the Lamarckian Genetic Algorithm (LGA) scoring function with the number of GA runs = 100, population size = 550, and a maximum number of evaluations = 24,000,000.

### Molecular dynamics simulation (MD-simulation) and free energy landscape (FEL) analysis

The MD simulations studies were carried out in triplicate on dock complexes for BACE1 (PDB I.D: 2ZHV) with FDB017657 using the Desmond 2020.1 from Schrödinger, LLC. The triplicate samplings were made using the same parameters for each MD run to obtain the reproducibility of the results. The OPLS-2005 force field (Bowers et al., 2006; Chow et al., 2008; Shivakumar et al., 2010) and explicit solvent model with the stocktickerSPC water molecules were used in this system (Jorgensen et al., 1983). Na^+^ ions were added to neutralize the charge of 0.15 M, and NaCl solutions were added to the system to simulate the physiological environment. Initially, the system was equilibrated using an NVT ensemble for 150 ns to retrain over the protein- FDB017657 complex. Following the previous step, a short run of equilibration and minimization was carried out using an NPT ensemble for 12 ns. The NPT ensemble was set up using the Nose-Hoover chain coupling scheme (Martyna et al., 1994) with the temperature at 27°C, the relaxation time of 1.0 ps, and pressure of 1 bar maintained in all the simulations. A time step of 2fs was used. The Martyna–Tuckerman–Klein chain coupling scheme (Martyna et al., 1992) barostat method was used for pressure control with a relaxation time of 2 ps. The particle mesh Ewald method (Toukmaji and Board, 1996) was used to calculate long-range electrostatic interactions, and the Radius for the Coulomb interactions was fixed at 9Å. RESPA integrator was used for a time step of 2 fs for each trajectory to calculate the bonded forces. The root means square deviation (RMSD), radius of gyration (Rg), root mean square fluctuation (RMSF), and the number of hydrogen (H-bonds) were calculated to monitor the stability of the MD simulations. The free energy landscape of protein folding on the FDB017657 bound complex was measured using geo_measures v 0.8 (Kagami et al., 2020). Geo_measures include a powerful library of g_sham and form the MD trajectory against RMSD and Radius of gyration (Rg) energy profile of folding recorded in a 3D plot using matplotlib python package.

### Molecular mechanics generalized born and surface area (MMGBSA) calculations

During MD simulations of BACE1 complexed with FDB017657, the binding free energy (Gbind) of docked complexes was calculated using the premier molecular mechanics generalized Born surface area (MM-GBSA) module (Schrodinger suite, LLC, New York, NY, United States, 2017-4). The binding free energy was calculated using the OPLS 2005 force field, VSGB solvent model, and rotamer search methods (Piao et al., 2019). After the MD run, 10 ns intervals were used to choose the MD trajectories frames. The total free energy binding was calculated using equation 1:


(1) ΔGbind=Gcomplex-(Gprotein+Gligand)

Where, ΔGbind = binding free energy, Gcomplex = free energy of the complex, Gprotein = free energy of the target protein, and Gligand = free energy of the ligand. The MMGBSA outcome trajectories were analyzed further for post-dynamics structure modifications.

### Dynamic cross-correlation and principal component (PCA) analysis

During a 150 ns MD simulation, a dynamic cross-correlation matrix (DCCM) was constructed across all C-atoms for all complexes to examine domain correlations. During a 150 ns simulation of the BACE1 (PDB I.D- 2ZHV) complexed with FDB017657, PCA analysis was used to recover the global movements of the trajectories. To calculate the PCA, a covariance matrix was created as stated. For conformational analysis of the FDB017657 in bound complex, 20 alternative conformational modes of the main component as movements of trajectories were calculated, and a comparison of the first highest mode (PC2) with PC10 was investigated. Geo measures v 0.8 was used to calculate the free energy landscape of protein folding on an FDB017657-bound complex (Kagami et al., 2020). The MD trajectory versus PC2 and PC10 energy folding profiles were recorded in a 3D plot using the matplotlib python package using Geo measures, which includes a comprehensive library of g_sham.

## Results

The present QSAR analysis is performed using a moderate-size data set comprising structurally diverse compounds with experimentally measured Ki in the range from 0.47 to 1,400 nM. Thus, it covers a sufficiently broad chemical and data range. This helped to derive a properly validated (Martin and Muchmore, 2012; Gramatica et al., 2013; Masand et al., 2015; Fujita and Winkler, 2016) genetic algorithm unified with multilinear regression (GA-MLR) model to collect or extend thorough information about the pharmacophoric features that control the desired bio-activity (Descriptive QSAR) and having adequate external predictive capability (Predictive QSAR). The six variable-based GA-MLR QSAR model along with selected internal and external validation parameters (see Supplementary material for additional parameters) is as follows:

QSAR Model (Divided Set: Training Set-80% and Prediction Set-20%):

pKi = 4.415 (± 0.236) + 0.046 (± 0.017) * com_lipohyd_5A + 0.12 (± 0.027) * faccC3B + 0.353 (± 0.105) * aroC_sumpc + 0.273 (± 0.034) * N_acc_5B + 0.109 (± 0.02) * aroC_ringS_6B + 0.269 (± 0.04) * fsp3OringC8B +

Statistical parameters related to fitting, double cross-validation, and Y-scrambling for the *de novo* QSAR model with thresholds for some parameters (bottom of table) are shown in Table 1.

**TABLE 1:** Statistical parameters for the developed QSAR model.

Statistical parameters	Model
**Fitting**	
R^2^	0.8120
R^2^_adj_	0.8168
R^2^-R^2^_adj_	0.0037
LOF	0.1807
K_xx_	0.2382
Delta K	0.0928
RMSE_tr_	0.4079
MAE_tr_	0.3276
RSS_tr_	49.5888
CCC_tr_	0.9014
s	0.4128
F	221.7565
**Internal validation**	
Q^2^_LOO_	0.8120
R^2^-Q^2^_LOO_	0.0085
RMSE_cv_	0.4175
MAE_cv_	0.3352
PRESS_cv_	51.9415
CCC_cv_	0.8968
Q^2^_LMO_	0.8123
R^2^_Yscr_	0.0197
RMSE AV_Yscr_	0.9534
Q^2^*^Yscr^*	–0.0283
External validation	
RMSE_ext_	0.4604
MAEext	0.3803
PRESS_ext_	15.4724
R^2^_ext_	0.7829
Q^2^-_F1_	0.7832
Q^2^-_F2_	0.7819
Q^2^-_F3_	0.7714
CCC_ext_	0.8742
r^2^_m_ aver.	0.6607
r^2^_m_ delta	0.1977
k′	0.9967
K	0.9999
Clos′	0.0496
Clos	0.0000

Thresholds for some important statistical parameters: *R*^2^ ≥ 0.6, Q^2^_LOO_ ≥ 0.5, Q^2^_LMO_ ≥ 0.6, *R*^2^ > Q^2^, R^2^_ex_ ≥ 0.6, RMSE_tr_ < RMSE_cv_, ΔK ≥ 0.05, CCC ≥ 0.80, Q^2^_Fn_ ≥ 0.60, r^2^m ≥ 0.6, 0.9 ≤ k ≤ 1.1 and 0.9 ≤ k′ ≤ 1.1 at RMSE≈2, MAE 4 ≈04 R^2^_adj_ of fitting parameter R^2^, etc.) The threshold is significantly exceeded, confirming the adequacy of the number of molecular descriptors in the model and the statistical acceptability of the QSAR model. The values of Q^2^_LOO_, Q^2^_LMO_, etc., (internal validation parameters) confirm the statistical robustness of the QSAR model. The high values of the external test parameters R^2^_ex_, Q^2^_F1_, Q^2^_F2_, Q^2^_F3_, etc., emphasize the external predictability of the QSAR model. The coverage area of the model (Applicability Domain) is determined from Williams plots for the QSAR model (see Figure 3). Almost all statistical parameters reached values well above the accepted threshold, and the minimal correlation between the selected molecular descriptors precluded the possibility of random development of the QSAR model. This data confirms the statistical reliability and high external predictability of the developed QSAR models.

**FIGURE 3:** Graph for **(A)** experimental vs. predicted pKi **(B)** experimental vs. residuals **(C)** Williams plot for applicability domain **(D)** Insubria Plot.

A nicely proven correlation among salient capabilities of the molecules represented through molecular descriptors, and their bioactivity expands statistics approximately mechanistic elements of molecules, specificity, and quantity (presence or even absence) of various structural developments for preferred bioactivity. Although, withinside the QSAR analysis, we’ve as compared the Ki values of various molecules in correlation and as an impact of a specific molecular descriptor, a similar or contrary impact of different molecular descriptors or unknown descriptors has a dominant impact in figuring out the general Ki value of a molecule cannot be neglected. In different words, a single molecular descriptor is incapable of absolutely explaining the experimental Ki value for this sort of numerous set of molecules. That is, the successful usage of the advanced QSAR model is based on the concomitant usage of molecular descriptors.

### Mechanistic interpretation

com_lipohyd_5A (occurrence of the lipo-hydrophobic atoms within 5A from the center of mass of the molecule) Since this descriptor received a positive coefficient in the developed QSAR model, increasing the value of the molecular descriptor com_lipohyd_5A was observed to increase BACE1 inhibitory activity. This can be observed by comparing the compound 368 (pKi = 7.75, com_lipohyd_5A = 14) with 48 (pKi = 6.37, com_lipohyd_5A = 13) for which an increase in the value of the molecular descriptor com_lipohyd_5A from 13 for the molecule 48 to the 14 will give rise to increase in pKi value by about 1 unit (about ten-fold increase in BACE1 inhibitory activity). This observation is further reinforced by the following pair of molecules; 243 (pKi = 7.35, com_lipohyd_5A = 8) and 134 (pKi = 6.93, com_lipohyd_5A = 7), 211 (pKi = 7.92, com_lipohyd_5A = 12) and 207 (pKi = 7.58, com_lipohyd_5A = 11), 189 (pKi = 8.4, com_lipohyd_5A = 15) and 255 (pKi = 8.19, com_lipohyd_5A = 10), 262 (pKi = 5.52, com_lipohyd_5A = 15) and 115 (pKi = 4.97, com_lipohyd_5A = 13), etc. Shifting the molecular descriptor com_lipohyd_5A with com_lipohyd_6A statistically improves the performance (R: 0.84) of the developed QSAR model, while replacing com_lipohyd_5A with com_lipohyd_4A statistically drops the performance of the QSAR model (R: 0.81). This observation underscores the importance of the molecular descriptor com_lipohyd_5A. In addition, the optimum distance between lipo-hydrophobic atoms from the center of mass of the molecule should be maintained at 6 Å to show better inhibitory activity against BACE1.

faccC3B (occurrence of the carbon atom exactly at three bonds from the acceptor atom). If the same descriptor exists in two or four bonding at the same time, it will be removed during the calculation of faccC3B. This descriptor received a positive sign in the developed QSAR model. Therefore, further increases in faccC3B value increase the inhibitory efficacy of BACE1 inhibitors. Comparison of the compound 331 (pKi = 7.6, faccC3B = 7) with 142 (pKi = 6.87, faccC3B = 6) illustrate the influence of the molecular descriptor faccC3B. If the value of the molecular descriptor faccC3B is enhanced from 6 for the molecule 142 to 7 will upsurge the pki value by about 1 unit (about 10-fold amplification in the BACE1 inhibitory activity). Following pair from Figures 3C,D of molecules support this observation; 295 (pKi = 8.72, faccC3B = 6) and 255 (pKi = 8.19, faccC3B = 4), 262 (pKi = 5.52, faccC3B = 3) and 115 (pKi = 4.97, faccC3B = 2), 258 (pKi = 8.7, faccC3B = 9) and 274 (pKi = 7.58, faccC3B = 8), 128 (pKi = 6.28, faccC3B = 3) and 60 (pKi = 6.1, faccC3B = 2), 169 (pKi = 8.7, faccC3B = 9) and 286 (pKi = 7.55, faccC3B = 7), etc.

This shows that simple carbon atoms along the 3-bond acceptor atom are essential for inhibitory efficacy, but the molecular descriptors faccC3B and fdonC3B (frequency of carbon atoms exactly 3 bonds away from the donor atom). Or fdonlipo5B (an acceptor atom with exactly 5 bonds from the donor atom) greatly improves the statistical detection power of the developed QSAR model (fdonC3B, R: 0.89) (fdonlipo5B, R: 0.88). This observation shows that the inhibitory effect can be enhanced by replacing the acceptor atom with a donor atom with 3 bonds of the same topology distance, or by moving the carbon atom to any lipophilic atom along the donor by a distance of five bonds. This observation shows that the carbon atom is more important along the donor atom located at the optimum distance of the three bonds. Therefore, since most H-bond donors or acceptors are nitrogen or oxygen, the presence of donor atoms close to the carbon atom may help to enhance the interaction with the polar residues of the receptor (BACE1). In addition, the descriptor also shows the important role that carbon atoms definitely play in lipophilicity.

aroC_sumpc (sum of partial charges on aromatic carbon atoms in the range of + 0.2 and −0.2). A positive coefficient for aroC_sumpc indicates that the higher the value of this descriptor, the better the activity profile. The presence of a large number of carbon atoms makes the molecule lipophilic, while the presence of positively or negatively charged carbon atoms causes various types of hydrophobic interactions with the receptor (BACE1), such as pi-alkyl, pi-cation, and pi-pi stacking. This observation underscores the importance of the molecular descriptor aroC_sumpc. This observation is supported by comparing the following pairs of molecules: 316 (pKi = 8.5, aroC_sumpc = 0.224000013) and 23 (pKi = 7.4, aroC_sumpc = −0.088000003), 159 (pKi = 9, aroC_sumpc = 0.013999997) and 298 (pKi = 8.5, aroC_sumpc = −0.197999999), 369 (pKi = 9, aroC_sumpc = 0.356000006) and 109 (pKi = 8.14, aroC_sumpc = −0.32299999), etc. This observation pointed out that negatively charged carbons are not favorable for BACE1 inhibitory activity, hence, ring carbon atom with neutral or positively charged possesses a better BACE1 inhibitory activity.

Subsequently, shifting the molecular descriptor aroC_sumpc to the molecular descriptor ringC_sumpc (sum of partial charges of the ring carbon atom) for future drug optimization increases the statistical power (R: 0.88) of the developed QSAR model. Furthermore, assuming that the molecular descriptor aroC_sumpc is replaced with the molecular descriptor aroCminus_sumpc (sum of partial charges of negatively charged aromatic carbon atoms), this reduces the statistical power (R: 0.75) of the QSAR model. Therefore, incorporating the ring carbon atom (ringC_sumpc) is a better choice for future optimization of hits to the lead molecule for better inhibitory activity of BACE1.

N_acc_5B (occurrence of acceptor atom within 5 bonds from the nitrogen atom). The molecular descriptor N_acc_5B indicates that the acceptor atom is within the four bonds of the nitrogen atom. This molecular descriptor has a positive coefficient in the developed QSAR model, so increasing the number of such combinations can enhance BACE1 inhibition. The effect of N_acc_5B can be explained by comparing the molecule 258 (pKi = 8.7, N_acc_5B = 5) and 57 (pKi = 6.4, N_acc_5B = 3). For molecule 57, if the value of the molecule descriptor increase from 3 to 5 will further amplify the pKi value by about 2 units, therefore, enhancing the BACE1 inhibitory activity by about 20 folds. These descriptors pointed out the importance of the nitrogen atom in BACE1 inhibitory activity. Moreover, additional molecular pair also illustrate the effect of N_acc_5B on BACE1 inhibitory activity include; 250 (pKi = 7.64, N_acc_5B = 5) and 55 (pKi = 6.52, N_acc_5B = 3), 189 (pKi = 8.4, N_acc_5B = 5) and 252 (pKi = 7.57, N_acc_5B = 4), 297 (pKi = 8.0, N_acc_5B = 8) and 102 (pKi = 7.17, N_acc_5B = 7), 312 (pKi = 8.5, N_acc_5B = 4) and 213 (pKi = 6.2, N_acc_5B = 3), etc.

The shift of the molecular descriptor N_acc_5B by the molecular descriptor N_acc_2B (the occurrence of acceptor atoms within two bonds from the nitrogen atom) strongly affects the statistical performance (R: 0.86) of the developed QSAR model (N_don_5B). This observation shows that the subsequent descriptor is N_acc_2B, which is useful as a better alternative to future drug optimization and to enhance the BACE1 inhibitor activity. Again, it is suggested that the optimum distance between the acceptor atom and the nitrogen atom may be two bonds.

On the other hand, replacing the molecular descriptor N_acc_5B with the molecular descriptor N_don_5B (the appearance of a donor atom within 5 bonds from the nitrogen atom) significantly increases the statistical power (R: 0.85) of the developed QSAR model. This remark reveals two strategies for future optimization, consisting of reducing the topological distance from five bonds to two bonds according to the N_acc_2B descriptor, and replacement of acceptors with donors by maintaining the optimal distance of five bonds. This observation underscores the importance of nitrogen atoms and acceptor/donor properties for better inhibitory activity of BACE1.

aroC_ringS_6B (occurrence of the ring sulfur atoms within six bonds from the aromatic carbon atoms). The positive coefficient of the developed QSAR model descriptor justifies the increase in the value of the aroC_ringS_6B descriptor and further enhances the BACE1 inhibitory activity. Shifting the molecular descriptor aroC_ringS_6B by fringSringC3B (frequency of ring carbon atoms in exactly three bonds from the ring sulfur atom) significantly increases the statistical power (R:0.91) of the QSAR model. By comparing the molecule 222 (pKi = 8.0, aroC_ringS_6B = 1) and 362 (pKi = 7.75, aroC_ringS_6B = 0), the influence of aroC_ringS_6B as illustrated in the Figures 4A–J. Moreover, amplification in the value of the molecular descriptor aroC_ringS_6B from 0 to 1 for the molecule will uplift the pKi value by about 0.75 units (about 7 fold increase in the BACE1 inhibitory activity). Another pair of molecules also illustrate the effect of aroC_ringS_6B on BACE1 inhibitory activity include; 256 (pKi = 8.5, aroC_ringS_6B = 2) and 2 (pKi = 7.5, aroC_ringS_6B = 1), 295 (pKi = 8.7, aroC_ringS_6B = 2) and 324 (pKi = 7.3, aroC_ringS_6B = 0), 189 (pKi = 8.4, aroC_ringS_6B = 2) and 254 (pKi = 8.1, aroC_ringS_6B = 1), 144 (pKi = 7.8, aroC_ringS_6B = 2) and 140 (pKi = 7.0, aroC_ringS_6B = 0), etc.

**FIGURE 4:** **(A,B)** Depiction of molecular descriptor com_lipohyd_5A for the compound 368 and 48 (pink star in the in both molecules indicates center of mass of the molecule). **(C,D)** Depiction of molecular descriptor faccC3B for the compound 331 and 48. **(E,F)** Illustration of the molecular descriptor N_acc_5B for the molecule 258 and 57. **(G,H)** Presentation of the molecular descriptor aroC_ringS_6B for the molecule 222 and 362. **(I,J)** Illustration of molecular descriptor fsp3OringC8B for the molecule 362 and 48.

Furthermore, replacing the molecular descriptor aroC_ringS_6B with fringSringC5B (frequency of ring carbon atoms in exactly five bonds from the ring sulfur atom) shows an increase in the statistical power (r: 0.94) of the developed QSAR model. On the other hand, replacing the molecular descriptor aroC_ringS_6B with fringSC6B (frequency of carbon atoms appearing in exactly 6 bonds from the ring sulfur atom) significantly reduces the statistical power (R: 0.80) of the QSAR model. This observation emphasizes the importance of the ring carbon atom and the ring sulfur atom. Furthermore, it can be concluded that reducing the topology bond distance from six to five bonds strongly affects the inhibitory activity of BACE1. Therefore, in future drug designs, it is recommended to keep the optimal distance between the ring carbon and the ring sprue atom at five bonds in order to increase the inhibitory activity of base 1. Aromatic and heterocyclic rings are very powerful motifs in drug discovery with target proteins such as the classical arene-arene interactions (π stacking), π-sulfur interactions, and arene-cation interaction. It offers many unique and powerful interactions such as bonds (end-face interactions) and recently identified π cations.

fsp3OringC8B (frequency of occurrence of the ring carbon atom exactly at eight bonds from the sp3 oxygen atom) If the same ring carbon atom occurs simultaneously in seven or nine bonds, it will be bypassed in the fsp3OringC8B calculation. This molecular descriptor has a positive coefficient in the developed QSAR model, so increasing its value can improve the Ki value.

The effect of fsp3OringC8B can be assessed by comparing the molecule 362 9 (pKi = 7.75, fsp3OringC8B = 2) with 48 (pKi = 6.37, fsp3OringC8B = 1). Increasing the value of fsp3OringC8B for molecule 1 to 2 for molecule 48 will upsurge the pKi value by 1.38unit (about 13-fold amplification in the BACE1 inhibitory potential). Following pair of molecules also explain the effect of fsp3OringC8B on BACE1 inhibitory activity; 211 (pKi = 7.9, fsp3OringC8B = 3) and 207 (pKi = 7.5, fsp3OringC8B = 1), 299 (pKi = 8.7, fsp3OringC8B = 2) and 255 (pKi = 8.1, fsp3OringC8B = 1), 352 (pKi = 8.4, fsp3OringC8B = 2) and 30 (pKi = 6.0, fsp3OringC8B = 0), 110 (pKi = 7.5, fsp3OringC8B = 4) and 66 (pKi = 6.5, fsp3OringC8B = 0), etc. Replacing the fsp3OringC8B molecular descriptor with the fsp3OringC9B descriptor significantly reduces the statistical power (R: 0.78) of the developed QSAR model.

This observation underscores the importance of the molecular descriptor fsp3OringC8B. Therefore, future drug designs need to maintain the optimal distance between sp3 hybridized oxygen and ring carbon atoms at eight bonds in order to achieve better BACE1 inhibitory activity. Most oxygen atoms act as either acceptors or ether linkage, which can confer lipophilicity on the molecule. This may help to enhance both polar and hydrophobic interactions with the BACE1 receptor.

### Molecular docking for validation of docking score

In molecular docking analysis of the BACE1 with FDB017657 in Autodock output, a dock complex displayed the best conformation. Receptors and ligands were saved in the.pdbqt format for subsequent usage using the MGL 1.5.6 suite. Vina was launched from a command prompt using the command line. In the setup, the default grid point spacing was 0.525 and the exhaustiveness was set to 8. The output files were in.pdbqt format, and they were analyzed using PyMol and the Discovery studio visualizer 2021. The ligand-binding was validated and optimized using the co-crystal ligand. Both the receptor and ligands were made by combining 48 polar hydrogen bonds and detecting 1 rotatable bond and adding Kollman and Gasteiger charges. Finally, both receptor and ligand molecules were stored in the.pdbqt format. With the values *X* = −1.655, *Y* = 57.005, and *Z* = 133.83, a grid box was produced with a spacing of 0.375. Docking experiments of the protein-ligand complex were carried out using Genetic Algorithm (GA) parameters were set with 100, population size was made 300 with a maximum number of evaluates was set to low at 2,500,000 and maximum generations of 27,000. Further docking experiments of the protein–ligand complex were carried out using the Lamarckian Genetic Algorithm (LGA) to obtain the lowest free energy of binding (G). The 2ZHV-FDB017657 complex showed free energy of binding (ΔG) −8.9 kcal/mol, inhibitory concentration (Ki) 990.57 μM, ligand efficiency −1.26, total internal energy −1.45 kJ/mol, and torsional energy 0.3 kJ/mol. The docking scores are mentioned in Table 2.

**TABLE 2:** Screening of phytochemicals based on their best binding energy.

Protein-ligand	Binding affinity (kcal/mol)
2zhv_8265	−4.8
2zhv_8263	−4.7
2zhv_8262	−7.3
2zhv_8079	−4.7
2zhv_7888	−5
2zhv_7701	−6.4
2zhv_7594	−6.3
2zhv_7334	−2.9
2zhv_7032	−4.9
2zhv_6574	−5.1
2zhv_5179	−5.6
2zhv_4844	−7.6
2zhv_4817	−5.6
2zhv_4693	−4.9
2zhv_4688	−5.8
2zhv_4605	−5.5
2zhv_4468	−**8.9**
2zhv_4340	−7.6
2zhv_4009	−5.7
2zhv_3981	−4.6
2zhv_3805	−4.7
2zhv_3207	−5.7
2zhv_2839	−4.8
2zhv_1976	−5.4
2zhv_1749	−5.7
2zhv_734	−7.3
2zhv_686	−6.7
2zhv_673	−8.3
2zhv_603	−6.5
2zhv_442	−4.5
2zhv_41	−3.8
2zhv_4	−5.6

The principal residues making the binding pocket around 4-(3,4-dihydroxyphenyl)-2-hydroxy-1H-phenalen-1-one (Food I.D: FDB017657) are comprised of THR72, THR231, GLY230, ASP228, GLY34, ILE118, SER35, PHE108, ASP106, LYS107, GLY74, and GLN73 by Van der Waals interaction forces; ASP32 is involved in conventional hydrogen bonding, while TYR71 is involved in forming a conventional Pi-Pi bond (Figure 5, left).

**FIGURE 5:** Best docked pose of FDB017657 with 2ZHV displaying 2D interaction plot on the **left panel**. Pink dashed lines indicate the Pi-Alkyl bond and residues embedded in the light green sphere, indicating involvement in Van der Waals interactions. On the **center panel**, surface view of 2ZHV displays binding cavity of FDB017657, and **right panel** displays the zoomed-out binding pocket having amino acid residues at 3Å surrounding the FDB017657 molecule.

### Molecular dynamics simulation (MD) and free energy landscape analysis

Molecular dynamics and simulation (MD) studies were carried out to determine the stability and convergence of the 4-(3,4-Dihydroxyphenyl)-2-hydroxy-1H-phenalen-1-one (PubChem I.D: 4468; Food I.D: FDB017657) bound BACE1 (PDB I.D: 2ZHV) complex. Each simulation of 150 ns displayed stable conformation while comparing the root mean square deviation (RMSD) values.

The Root Mean Square Deviation (RMSD) is a metric for calculating the average change in the displacement of a group of atoms in relation to a reference frame. It is calculated for each and every frame of the trajectory. The RMSD for frame x is:


$$RMSD_{X}=\sqrt{\frac{1}{N}\sum_{i=1}^{N}\left(r_{i}^{\prime }\left(t_{X}\right)\right)-r_{i}\left(t_{ref}\right)){}^{2}}$$

where N is the number of atoms in the atom selection; t_ref_ is the reference time (the first frame is usually used as the reference and is treated as time *t* = 0); and where *r*′ is the position of the selected atoms after superimposing on the reference frame in frame *x*, where frame x is recorded at time *t*_x_. Every frame in the simulation trajectory is subjected to the same technique (Maiorov and Crippen, 1994).

For characterizing local changes along the protein chain, the Root Mean Square Fluctuation (RMSF) is useful. The RMSF for residue *i* is:


$$RMSF_{i}=\sqrt{\frac{1}{T}\sum_{t=1}^{T}<\left(r_{i}^{\prime }\left(t\right)\right)-r_{i}\left(t_{ref}\right)){}^{2}>}$$

The angle brackets indicate that the average of square distance is taken over the selection of atoms in the residue. where T is the trajectory time over which the RMSF is calculated, t_ref_ is the reference time, r_i_ is the position of residue I r′ is the position of atoms in residue I after superposition on the reference. Its simulation paths of Desmond were examined. MD trajectory analysis was used to calculate the root mean square deviation (RMSD), root mean square fluctuation (RMSF), and protein–ligand interactions. Protein RMSD: The graphs depict the evolution of a protein’s RMSD (left *Y*-axis). The RMSD is estimated based on the atom selection once all protein frames are aligned on the reference frame backbone.

The Cα-backbone of BACE1 bound to 4-(3,4-dihydroxyphenyl)-2-hydroxy-1H-phenalen-1-one (PubChem I.D: 4468; Food I.D: FDB017657) exhibited a deviation of 0.4 Å (Figure 6A). RMSD plots are within the acceptable range signifying the stability of proteins in the FDB017657 bound state before and after simulation and it can also be suggested that FDB017657 bound BACE1 (PDB I.D: 2ZHV) is quite stable in the complex might be due to significant binding of the ligand.

**FIGURE 6:** **(A)** MD simulation trajectory analysis of Root Mean Square Divisions (RMSD) of FDB017657 bound with 2ZHV, i.e., BACE1 150 ns time frame in triplicate displayed: R1 (replicate 1) RMSD plot of FDB017657 bound BACE1 (PDB I.D: 2ZHV) (red) with control protein BACE1 (PDB I.D: 2ZHV) (light green); R2 (replicate 2) RMSD plot of FDB017657 bound BACE1 (PDB I.D: 2ZHV) (dark maroon) with control protein BACE1 (PDB I.D: 2ZHV) (juniper green); R3 (replicate 3) RMSD plot of FDB017657 bound BACE1 (PDB I.D: 2ZHV) (lemon yellow) with control protein BACE1 (PDB I.D: 2ZHV) (cyan). **(B)** MD simulation trajectory analysis of Root Mean Square Fluctuations (RMSF) of FDB017657 bound with BACE1 (PDB I.D: 2ZHV) at 150 ns time frame in triplicate displayed: R1 (replicate 1) RMSF plot of FDB017657 bound BACE1 (PDB I.D: 2ZHV) (navy blue) with control protein BACE1 (PDB I.D: 2ZHV) (black); R2 (replicate 2) RMSF plot of FDB017657 bound BACE1 (PDB I.D: 2ZHV) (canary yellow) with control protein BACE1 (PDB I.D: 2ZHV) (red); R3 (replicate 3) RMSF plot of FDB017657 bound BACE1 (PDB I.D: 2ZHV) (gray) with control protein BACE1 (PDB I.D: 2ZHV) (purple). **(C)** MD simulation trajectory analysis of Radius of gyration (Rg) of FDB017657 bound with BACE1 (PDB I.D: 2ZHV) at 150 ns time frame in triplicate displayed: R1 (replicate 1) Rg plot of FDB017657 bound BACE1 (PDB I.D: 2ZHV) (red) with control protein BACE1 (PDB I.D: 2ZHV) (light green); R2 (replicate 2) Rg plot of FDB017657 bound BACE1 (PDB I.D: 2ZHV) (dark maroon) with control protein BACE1 (PDB I.D: 2ZHV) (juniper green); R3 (replicate 3) Rg plot of FDB017657 bound BACE1 (PDB I.D: 2ZHV) (cyan) with control protein BACE1 (PDB I.D: 2ZHV) (lemon yellow). **(D)** MD simulation trajectory analysis of Hydrogen Bonding (H-Bonds) of FDB017657 bound with BACE1 (PDB I.D: 2ZHV) at 150 ns time frame in triplicate displayed: R1 (replicate 1) H-Bond plot of FDB017657 bound BACE1 (PDB I.D: 2ZHV) (red); R2 (replicate 2) H-Bond plot of FDB017657 bound BACE1 (PDB I.D: 2ZHV) (black); R3 (replicate 3) H-Bond plot of FDB017657 bound BACE1 (PDB I.D: 2ZHV) (light green).

The radius of gyration is the measure of the compactness of the protein. FDB017657 bound proteins displayed a lowering of radius of gyration (Rg) (Figure 6B; R1, R2, R3). The lowering of Rg indicates the compactness of the protein–ligand complex. From the overall quality analysis from RMSD and Rg, it can be suggested that FDB017657 bound to the protein targets posthumously in the binding cavities and plays a significant role in the stability of the proteins.

The plots for root mean square fluctuations (RMSF) displayed a significant RMSF in BACE1 protein at a few residues at the specific time function of 150 ns. Peaks show sections of the protein that fluctuate the greatest during the simulation on the RMSF plot. Typically, the tails (N- and C-terminal) of proteins change more than any other portion of the protein. Secondary structural parts such as alpha helices and beta strands are usually more rigid than the unstructured portion of the protein and fluctuate less than loop areas. The residues with higher peaks belong to loop areas or N and C-terminal zones, as determined by MD trajectories (Figure 6C). The stability of ligand binding to the protein is shown by low RMSF values of binding site residues. From the triplicate runs of BACE1, as shown in Figure 6C, a few fluctuating peaks can be seen although mostly the complex is found to be stabilized as shown in Figure 6C. The RMSF values are acceptable for stabilizing the protein–ligand complex. Therefore, in RMSF plots, it can be suggested that the protein structures were stable during simulation in FDB017657 bound conformation.

The average hydrogen bonds formed between FDB017657 and the respective protein, BACE1 (PDB I.D: 2ZHV), during the 150 ns simulation were also recorded (Figure 6D). From 0 ns to 150 ns a formation of hydrogen bonding was found throughout the simulation and the same for triplicate MD simulation of FDB017657 with BACE1 (Figure 6D). Moreover, the pattern of two hydrogen bond formation with BACE1 (PDB I.D: 2ZHV), in docking was corroborated by the number of hydrogen plot analyses after 150 ns molecular dynamics (Figure 6D). The amount of hydrogen bonds between BACE1 with FDB017657 has strengthened the binding and facilitated to conform to a more stable complex during the simulation.

Throughout the simulation, protein interactions with the ligand can be observed. As seen in the graph above, these interactions can be classified and summarized by type. Hydrogen bonds, hydrophobic, ionic, and water bridges are the four forms of protein–ligand interactions (or “contacts”). Each interaction type has a number of subtypes that can be examined using Maestro’s “Simulation Interactions Diagram” panel (see Figure 7A). The stacked bar charts are standardized over the course of the trajectory. Some protein residues may make several interactions of the same subtype with the ligand, values above 1.0 are feasible. As shown in Figure 7A, the majority of the significant ligand–protein interactions discovered by MD are hydrogen bonds and hydrophobic interactions. For 2ZHV- FDB017657, complex residues VAL_31, ASP_32, TYR_71, and THR_72 are the most important ones in terms of H-bonds.

**FIGURE 7:** **(A)** Protein-ligand contact histogram (H-bonds, Hydrophobic, Ionic, Water bridges) of the ligand, FDB017657 bound with 2ZHV recorded in a 150 ns simulation interval. **(B)** Ligand atom interactions with the protein residues of 2ZHV bound with FDB017657. **(C)** Secondary Structure element distribution by residue index throughout the protein structure. Red indicates alpha helices, and blue indicate beta-strands of 2ZHV bound with FDB017657. **(D)** Ligand torsion profile.

Individual ligand atom interactions with protein residues are depicted in Figure 7B. Interactions that occur for more than 30.0% of the simulation period in the chosen trajectory (0.00 through 150.0 ns) are displayed. From Figure 7B, it can be concluded that the amino acid residues: PHE108, TRP76, TYR71, and VAL69 involve a hydrophobic interaction, LYS107, ARG128 possess a positive charge bonding with the ligand, GLN73, SER35, and ASN37 are involved in polar interactions, and ASP32 and ASP228 are involved in negatively charged interaction with the ligand, FDB017657 in 150 ns simulation time scale.

Throughout the simulation, the existence of protein secondary structural elements (SSE) such as alpha helices and beta strands is examined to ensure that they are not present. The plot shown in Figure 7C depicts the distribution of SSE by residue index over the complete protein structure, and it encompasses the full protein structure. In contrast to the charts, which show the summary of the SSE composition for each trajectory frame during the course of the simulation, the graphs at the bottom show the evolution of each residue and its SSE assignment throughout the experiment. Throughout the simulation, alpha-helices and beta-strands are monitored as secondary structure elements (SSE). The left graph shows the distribution of SSE across the protein structure by the residue index. The top image highlights the SSE composition for each trajectory frame throughout the simulation, while the bottom plot tracks each residue’s SSE assignment through time.

It can be observed from Figure 7D, how each rotatable bond (RB) in the ligand alters its conformation throughout the simulation on the ligand torsions map (0.00 through 150.15 ns). The top panel shows a two-dimensional schematic of a ligand with color-coded rotatable bonds. There includes a dial plot as well as bar plots in the same color for each rotatable bond torsion. The evolution of the torsion’s conformation during the simulation is depicted using dial (or radial) graphs. The simulation’s time evolution is depicted radially outwards from the simulation’s start point at the center of the radial plot. The data from the dial plots are summarized in the bar plots, which show the torsion probability density in the data. Alternatively, if torsional potential data is available, the graphic will also indicate the rotatable bond’s potential (by summing the potential of the related torsions) kcal/mol. The potential values are given as kcal/mol and plotted on the graph’s left *Y*-axis. The histogram and torsion potential correlations can reveal the conformational strain that the ligand is under in order to maintain a protein-bound conformational state.

The stepwise trajectory analysis of every 25 ns of simulation of FDB017657 with BACE1 displayed the positional alteration with reference to the 0 ns structure (Figure 8). It has been observed that the ligand, FDB017657 has possessed a structural angular movement at the end frame to achieve its conformational stability and convergence.

**FIGURE 8:** Stepwise trajectory analysis for every 25 ns displaying the protein, BACE1 (PDB I.D: 2ZHV) and ligand conformation during 150 ns of simulation of 4-(3,4-Dihydroxyphenyl)-2-hydroxy-1H-phenalen-1-one (PubChem I.D: 4468; Food I.D: FDB017657).

The free energy landscape (FEL) of achieving global minima of Cα backbone atoms of proteins with respect to RMSD and radius of gyration (Rg) is displayed in Figure 9, BACE1 bound to the ligand, FDB017657 achieved the global minima (lowest free energy state) at 1.1 Å and Rg 20.9 Å (Figure 9). The FEL envisaged a deterministic behavior of BACE1 to the lowest energy state owing to its high stability and best conformation at FDB017657 bound state.

**FIGURE 9:** Free Energy Landscape displaying the achievement of global minima (ΔG, kJ/mol) of BACE1 in presence of FDB017657 with respect to their RMSD (nm) and Radius of gyration (Rg, nm).

### Molecular mechanics generalized born and surface area calculations

To assess the binding energy of ligands to protein molecules, the MMGBSA technique is commonly employed. The binding free energy of each BACE1– FDB017657 complex, as well as the impact of other non-bonded interaction energies, were estimated. With BACE1, the ligand FDB017657 has a binding energy of −53.4670 kcal/mol. Non-bonded interactions like G_bind_Coulomb, G_bind_Covalent, G_bind_Hbond, G_bind_Lipo, G_bind_SolvGB, and G_bind_vdW govern Gbind. Across all types of interactions, the G_bind_vdW, G_bind_Lipo, and G_bind_Coulomb energies contributed the most to the average binding energy. On the other side, the G_bind_SolvGB and Gbind Covalent energies contributed the least to the final average binding energies. Furthermore, the G_bind_Hbond interaction values of BACE1–FDB017657 complexes demonstrated stable hydrogen bonds with amino acid residues. In all of the compounds, G_bind_SolvGB and G_bind_Covalent exhibited unfavorable energy contributions and so opposed binding. Figure 10 (left panel) reveals that between pre-simulation (0 ns) and post-simulation (0 ns), FDB017657 in the binding pocket of BACE1 has undergone a large angular change in the pose (curved to straight) (150 ns). These conformational changes lead to better binding pocket acquisition and interaction with residues, which leads to enhanced stability and binding energy (mentioned in Table 3).

**FIGURE 10:** MMGBSA trajectory (0 ns, before simulation and 150 ns, after simulation) exhibited conformational changes of FDB017657 upon binding with the protein 2ZHV. The arrows indicate the overall positional variation (movement and pose) of FDB017657 at the binding site cavity.

**TABLE 3:** Binding energy calculation of FDB017657 with 2ZHV and non-bonded interaction energies from MMGBSA trajectories.

Energies (kcal/mol)	2ZHV
ΔG_bind_	−53.467 ± 3.001
ΔG_bind_Lipo	−22.124 ± 2.448
ΔG_bind_vdW	33.667 ± 0.0701
ΔG_bind_Coulomb	−9.827 ± 5.083
ΔG_bind_H_bond_	−1.465 ± 0.775
ΔG_bind_SolvGB	−8.989 ± 1.695
ΔG_bind_Covalent	−1.079 ± 1.049

Thus, MM-GBSA calculations resulted from MD simulation trajectories well justified with the binding energy obtained from docking results; moreover, the last frame (150 ns) of MMGBSA displayed the positional change of FDB017657 as compared to the 0 ns trajectory signifying the better binding pose for best fitting in the binding cavity of the protein (see Figure 10).

Therefore, it can be suggested that the FDB017657 molecule has a good affinity for the major target BACE1.

### Dynamic cross-correlation, principal component analysis (PCA), and energy calculations

Molecular dynamics simulation trajectories are analyzed for dynamic cross-correlation among the domains within protein chains bound with the FDB017657 molecule. For correlative dynamic motion, the cross-correlation matrices of BACE1 were generated and displayed in Figure 11. The blue blocks displayed in the figure indicated the residues having high correlated movement and red having the least correlation. The amino acid residues of FDB017657 bound BACE1 showed the concerted movement of residues (Figure 11).

**FIGURE 11:** Dynamic Cross Correlation matrix (DCCM) of 2ZHV and correlated amino acids conformed into secondary structural domains (colored) and non-correlated domains (gray) of 2ZHV.

Principal component analysis (PCA) determines the relationship between statistically meaningful conformations (major global motions) sampled during the trajectory. PCA of the MD simulation trajectories for BACE1 bound to the FDB017657 molecule was analyzed to interpret the randomized global motion of the atoms of amino acid residues. The internal coordinates mobility into three-dimensional space in the spatial time of 150 ns were recorded in a covariance matrix and the rational motion of each trajectory is interpreted in the form of orthogonal sets or Eigen vectors. In the BACE1 trajectory, PCA indicates statistically significant conformations. It is possible to identify the major motions within the trajectory as well as the critical motions required for conformational changes. In BACE1 bound to FDB017657, two different clusters along the PC1 and PC2 planes are exhibited that indicate a non-periodic conformational shift (Figure 12A). While these global motions are periodic because the groupings along the PC3 and PC4 planes do not totally cluster separately (Figure 12B). Moreover, a high periodic global motion was observed along the PC9 and PC10 planes due to the grouping of trajectories in a single cluster at the center of the PCA plot (Figure 12C). Centering of the trajectories in a single cluster indicates the periodic motion of MD trajectories due to stable conformational global motion.

**FIGURE 12:** **(A)** PCA of 2ZHV- FDB017657 showing a stable configuration. **(B)** Energy plot of protein BACE1 and FDB017657 complex system during the entire simulation event of 150 ns. **(C,D)** The change in PCA movements. The total energy (dark green), van der Waal’s energy (cyan) and Coulomb energy (red) of the entire system indicate the stability of the individual systems bound to FDB017657 molecule.

The energy profiles of the protein, BACE1 and FDB017657 complex systems, were determined to display the stability of the entire system. In this regard, the total energy (ETOT) of the BACE1 bound FDB017657 system was shown to be very stable with an average total energy of −69.00 kcal/mol (green). However, van der Waal’s energy (vdW) displayed to be merged over the total energy with an average energy of −40.00 kcal/mol and contemplated as a principal contributor to the stability of the BACE1-FDB017657 complex (cyan). In addition, Coulombic interactions played a minor role in the system stability and contributed to an average energy of −32.00 kcal/mol (red), (see Figure 12D).

## Discussion

Proteolytic processing of APP by BACE1 is the rate-determining step in Aβ production, hence BACE1 is employed as a therapeutic target for creating innovative lead compounds in AD in this study. According to the earlier reports, it was suggested that the enzyme BACE1 is also associated with different types of cancers and viruses in conjunction with AD. In this study, we have tried to reveal the potential of naturally available food molecules to bind the BACE1’s active site in a highly specific binding pattern. The aim of our study is toward the development of a drug from food compounds with the help of computational biology as it has the additional advantage regarding safety, and lesser chance of side effects. The low toxicity profile of natural products inspired by small-molecule inhibitors may prove to be a great asset during the frenetic development period of drug discovery when time is of the essence. Current state-of-the-art computational approaches can be used to identify structural and pharmacophoric properties of active natural compounds that can be used as drugs. Our results suggest that the selected 8,453 compounds from the Food database are majorly phenols and naphthol metabolites having a high potential of showing inhibitory activity against BACE1. The Food database is a recent database that proved the potential of food metabolites that we use in our daily life and found its major application in developing different therapeutics treating depressive disorders and others.

A nicely proven correlation among salient capabilities of the molecules represented through molecular descriptors, and their bioactivity expands statistics approximately mechanistic elements of molecules, specificity, and quantity (presence or even absence) of various structural developments for preferred bioactivity. Although, with the QSAR analysis, we’ve compared the Ki values of various molecules in correlation and as an impact of a specific molecular descriptor, a similar or contrary impact of different molecular descriptors or unknown descriptors has a dominant impact in figuring out the general Ki value of a molecule can’t be neglected. In other words, a single molecular descriptor is incapable of absolutely explaining the experimental Ki value for this sort of numerous sets of molecules. That is, the successful usage of the advanced QSAR model is based on the concomitant usage of molecular descriptors.

A QSAR model with multiple chemical descriptors is built using a dataset of 371 compounds. The resulting model was rigorously verified for fitting and internal validation to prove its strong external prediction capacity and resilience. In addition, virtual screening using QSAR yielded a novel food molecule with a better Ki value of 10.715 nM. Combined QSARs and molecular docking studies offered complimentary information and helped discover prodigious and under-privileged chemical characteristics that might be leveraged to change a molecule to produce better BACE1 inhibitors with higher Ki values. In the future, structural modifications that result in augmented values for the molecular descriptors with positive coefficients in the developed model for the anti-BACE1 activity will be performed to generate novel hits suitable for construction and *in vitro* evaluation as anti-Alzheimer’s (AD) disease therapy. These reports already demonstrated the potential of this plant as a source of novel drugs, nutraceuticals, and functional foods. Our present study perhaps supports a further avenue for *in vivo* and clinical trial of the food molecule, 4-(3,4-dihydroxyphenyl)-2-hydroxy-1H-phenalen-1-one to target BACE1 for any future scope to treat the AD along with viruses and cancer.

## Data availability statement

The original contributions presented in this study are included in the article/Supplementary material, further inquiries can be directed to the corresponding authors.

## Author contributions

NM and ADa performed the concept design. NM, AG, SwM, and RJ designed and carried out the experimental procedures. NM, AG, RJ, RB, MC, and VM done the analysis. NM, ADa, PD, AP, GM, SB, BA, and SA-H done the manuscript preparation. NM, ADe, GM, MK, AAl, ADa, SuM, AMA, and MZ edited the manuscript. All authors contributed to the article and approved the submitted version.

## Footnotes

1
https://www.ebi.ac.uk/chembl/g/#search_results/all/querybace1

2
www.acdlabs.com

3
http://foodb.ca/

4
https://www.rcsb.org/structure/2ZHV

## Supplementary material

Supplementary Table 1 Smileskipki.

Supplementary Table 2 Descriptor used in QSAR.

Supplementary Table 3 Formulas for calculation of model parameters.

Supplementary Table 4 Food molecules predicted pki and descriptors.

## References

[B1] Alzheimer’s Association (2012). 2012 Alzheimer’s disease facts and figures. *Alzheimer’s Dement.* 8 131–168.2240485410.1016/j.jalz.2012.02.001

[B2] ArifN.SubhaniA.HussainW.RasoolN. (2020). In silico inhibition of BACE-1 by selective phytochemicals as novel potential inhibitors: Molecular docking and DFT studies. *Curr. Drug Disc. Technol.* 17 397–411. 10.2174/1570163816666190214161825 30767744

[B3] BellacasaR. P.KarachaliouN.Estrada-TejedorR.TeixidóJ.CostaC.BorrellJ. I. A. L. K. (2013). and ROS1 as a joint target for the treatment of lung cancer: A review. *Transl. Lung Cancer Res.* 2 72–86.2580621810.3978/j.issn.2218-6751.2013.03.1PMC4369855

[B4] BermanH. M.WestbrookJ.FengZ.GillilandG.BhatT. N.WeissigH. (2000). The protein data bank. *Nucleic Acids Res.* 28 235–242. 10.1093/nar/28.1.235 10592235PMC102472

[B5] BoQ.RunhuaL.HanqingW.MinW.WenpengL.JinlunX. (2000). Chemical constituents from Musella lasiocarpa (Franch.) CY Wu. *Nat. Product Res. Develop.* 12 41–44.

[B6] BonvinoN. P.LiangJ.McCordE. D.ZafirisE.BenettiN.RayN. B. (2018). OliveNet™: A comprehensive library of compounds from Olea europaea. *Database* 2018:bay016. 10.1093/database/bay016 29688352PMC5808783

[B7] BowersK. J.ChowD. E.XuH.DrorR. O.EastwoodM. P.GregersenB. A. (2006). “Scalable algorithms for molecular dynamics simulations on commodity clusters,” in *SC’06: Proceedings of the 2006 ACM/IEEE Conference on Supercomputing*, (Tampa, FL: IEEE), 43–43. 10.1109/SC.2006.54

[B8] ChowE.RendlemanC. A.BowersK. J.DrorR. O.HughesD. H.GullingsrudJ. (2008). *Desmond performance on a cluster of multicore processors.* New York, NY: DE Shaw Research Technical Report DESRES/TR–2008-01.

[B9] CuiH.HungA. C.KlaverD. W.SuzukiT.FreemanC.NarkowiczC. (2011). Effects of heparin and enoxaparin on APP processing and aβ production in primary cortical neurons from Tg2576 mice. *PLoS One* 6:e23007. 10.1371/journal.pone.0023007 21829577PMC3146518

[B10] DaviesM.NowotkaM.PapadatosG.DedmanN.GaultonA.AtkinsonF. (2015). ChEMBL web services: Streamlining access to drug discovery data and utilities. *Nucleic Acids Res.* 45 D945–D954. 10.1093/nar/gkv352 25883136PMC4489243

[B11] De StrooperB.KarranE. (2016). The cellular phase of Alzheimer’s disease. *Cell* 164 603–615. 10.1016/j.cell.2015.12.056 26871627

[B12] DingwallC. (2001). Spotlight on BACE: The secretases as targets for treatment in Alzheimer disease. *J. Clin. Invest.* 108 1243–1246. 10.1172/JCI14402 11696563PMC209454

[B13] DongL. B.HeJ.LiX. Y.WuX. D.DengX.XuG. (2011). Chemical constituents from the aerial parts of Musella lasiocarpa. *Nat. Products Bioprospect.* 1 41–47. 10.1007/s13659-011-0007-7

[B14] ForliS.HueyR.PiqueM. E.SannerM. F.GoodsellD. S.OlsonA. J. (2016). Computational protein–ligand docking and virtual drug screening with the AutoDock suite. *Nat. Protocols* 11 905–919. 10.1038/nprot.2016.051 27077332PMC4868550

[B15] FujitaT.WinklerD. A. (2016). Understanding the Roles of the “Two QSARs”. *J. Chem. Inf. Model* 56 269–274. 10.1021/acs.jcim.5b00229 26754147

[B16] FukumotoH.CheungB. S.HymanB. T.IrizarryM. C. (2002). β-Secretase protein and activity are increased in the neocortex in Alzheimer disease. *Arch. Neurol.* 59 1381–1389. 10.1001/archneur.59.9.1381 12223024

[B17] GramaticaP. (2013). On the development and validation of QSAR models. *Methods Mol. Biol.* 930 499–526. 10.1007/978-1-62703-059-5_2123086855

[B18] GramaticaP. (2020). Principles of QSAR Modeling. *Int. J. Quant. Struct. Property Relation.* 5 61–97. 10.4018/IJQSPR.20200701.oa1

[B19] GramaticaP.CassaniS.ChiricoN. (2014). QSARINS-Chem: Insubria Datasets and New QSAR/QSPR Models for Environmental Pollutants in QSARINS. *J. Comput. Chem. Softw. News Updates* 35 1036–1044. 10.1002/jcc.23576 24599647

[B20] GramaticaP.ChiricoN.PapaE.KovarichS.CassaniS. (2013). QSARINS: A New Software for the Development, Analysis, and Validation of QSAR MLR Models. *J. Comp. Chem. Softw. News Updates* 34 2121–2132. 10.1002/jcc.23361

[B21] HallA.PekkalaT.PolvikoskiT.Van GilsM.KivipeltoM.LötjönenJ. (2019). Prediction models for dementia and neuropathology in the oldest old: The Vantaa 85+ cohort study. *Alzheimer’s Res. Ther.* 11 1–2. 10.1186/s13195-018-0450-3 30670070PMC6343349

[B22] HassanM.ShahzadiS.SeoS. Y.AlashwalH.ZakiN.MoustafaA. A. (2018). Molecular docking and dynamic simulation of AZD3293 and solanezumab effects against BACE1 to treat Alzheimer’s disease. *Front. Comput. Neurosci.* 12:34. 10.3389/fncom.2018.00034 29910719PMC5992503

[B23] HussainI.PowellD. J.HowlettD. R.ChapmanG. A.GilmourL.MurdockP. R. (2000). ASP1 (BACE2) cleaves the amyloid precursor protein at the β-secretase site. *Mol. Cell. Neurosci.* 16 609–619. 10.1006/mcne.2000.0884 11083922

[B24] JabirN. R.RehmanM. T.AlsolamiK.ShakilS.ZughaibiT. A.AlserihiR. F. (2021). Concatenation of molecular docking and molecular simulation of BACE-1, γ-secretase targeted ligands: In pursuit of Alzheimer’s treatment. *Ann. Med.* 53 2332–2344. 10.1080/07853890.2021.2009124 34889159PMC8667905

[B25] JawarkarR. D.BakalR. L.ZakiM. E. A.Al-HussainS.GhoshA.GandhiA. (2022). QSAR based virtual screening derived identification of a novel hit as a SARS CoV-229E 3CLpro Inhibitor: GA-MLR QSAR modeling supported by molecular Docking, molecular dynamics simulation and MMGBSA calculation approaches. *Arab. J. Chem.* 15:103499. 10.1016/j.arabjc.2021.103499 34909066PMC8524701

[B26] JorgensenW. L.ChandrasekharJ.MaduraJ. D.ImpeyR. W.KleinM. L. (1983). Comparison of simple potential functions for simulating liquid water. *J. Chem. Phys.* 79 926–935. 10.1063/1.445869

[B27] KagamiL. P.das NevesG. M.TimmersL. F. S. M.CaceresR. A.Eifler-LimaV. L. (2020). Geo-Measures: A Pymol plugin for protein structure ensembles analysis. *Comp. Biol. Chem.* 87:107322. 10.1016/j.compbiolchem.2020.107322 32604028

[B28] KimS.ChenJ.ChengT.GindulyteA.HeJ.HeS. (2019). PubChem 2019 update: Improved access to chemical data. *Nucleic Acids Res.* 47 D1102–D1109. 10.1093/nar/gky1033 30371825PMC6324075

[B29] LiQ.SüdhofT. C. (2004). Cleavage of amyloid-β precursor protein and amyloid-β precursor-like protein by BACE 1. *J. Biol. Chem.* 279 10542–10550. 10.1074/jbc.M310001200 14699153

[B30] LinX.KoelschG.WuS.DownsD.DashtiA.TangJ. (2000). Human aspartic protease memapsin 2 cleaves the β-secretase site of β-amyloid precursor protein. *Proc. Natl. Acad. Sci.* 97 1456–1460. 10.1073/pnas.97.4.1456 10677483PMC26455

[B31] MaiorovV. N.CrippenG. M. (1994). Significance of root-mean-square deviation in comparing three-dimensional structures of globular proteins. *J. Mol. Biol.* 235 625–634. 10.1006/jmbi.1994.1017 8289285

[B32] MartinY. C.MuchmoreS. W. (2012). Frozen out: Molecular modeling in the age of cryocrystallography. *J. Comput. Aided Mol. Design* 26, 91–92.10.1007/s10822-011-9537-722198477

[B33] MartynaG. J.KleinM. L.TuckermanM. (1992). Nosé–Hoover chains: The canonical ensemble via continuous dynamics. *J. Chem. Phys.* 97 2635–2643. 10.1063/1.463940

[B34] MartynaG. J.TobiasD. J.KleinM. L. (1994). Constant pressure molecular dynamics algorithms. *J. Chem. Phys.* 101 4177–4189. 10.1063/1.467468

[B35] MasandV. H.MahajanD. T.AlafeefyA. M.BukhariS. N.ElsayedN. N. (2015). Optimization of antiproliferative activity of substituted phenyl 4-(2-oxoimidazolidin-1-yl) benzenesulfonates: QSAR and CoMFA analyses. *Eur. J. Pharm. Sci*. 77, 230–237.2606641210.1016/j.ejps.2015.06.001

[B36] MasandV. H.RastijaV. (2017). PyDescriptor : A new PyMOL plugin for calculating thousands of easily understandable molecular descriptors. *Chemom. Intell. Labor. Syst.* 169 12–18. 10.1016/j.chemolab.2017.08.003

[B37] MorrisG. M.HueyR.LindstromW.SannerM. F.BelewR. K.GoodsellD. S. (2009). AutoDock4 and AutoDockTools4: Automated docking with selective receptor flexibility. *J. Comp. Chem.* 30 2785–2791. 10.1002/jcc.21256 19399780PMC2760638

[B38] Moussa-PachaN. M.AbdinS. M.OmarH. A.AlnissH.Al-TelT. H. (2020). BACE1 inhibitors: Current status and future directions in treating Alzheimer’s disease. *Med. Res. Rev.* 40 339–384. 10.1002/med.21622 31347728

[B39] MukerjeeN.DasA.MaitraS.GhoshA.KhanP.AlexiouA. (2022). Dynamics of natural product lupenone as a potential fusion inhibitor against the spike complex of novel semliki forest virus. *PLoS One* 17:e0263853. 10.1371/journal.pone.0263853 35213606PMC8880844

[B40] MurphyM. P.LeVineIII. H. (2010). Alzheimer’s disease and the amyloid-beta peptide. *J. Alzheimers Dis*. 19, 311–323. 10.3233/JAD-2010-1221 20061647PMC2813509

[B41] MusiN.ValentineJ. M.SickoraK. R.BaeuerleE.ThompsonC. S.ShenQ. (2018). Tau protein aggregation is associated with cellular senescence in the brain. *Aging cell* 17:e12840. 10.1111/acel.12840 30126037PMC6260915

[B42] NevesB. J.BragaR. C.Melo-FilhoC. C.Moreira-FilhoJ. T.MuratovE. N.AndradeC. H. (2018). QSAR-Based Virtual Screening: Advances and Applications in Drug Discovery. *Front. Pharmacol.* 9:1275. 10.3389/fphar.2018.01275 30524275PMC6262347

[B43] O’BoyleN. M.BanckM.JamesC. A.MorleyC.VandermeerschT.HutchisonG. R. (2011). Open Babel: An open chemical toolbox. *J. Cheminform.* 3:33. 10.1186/1758-2946-3-33 21982300PMC3198950

[B44] PettersenE. F.GoddardT. D.HuangC. C.CouchG. S.GreenblattD. M.MengE. C. (2004). UCSF Chimera—a visualization system for exploratory research and analysis. *J. Comp. Chem.* 25 1605–1612. 10.1002/jcc.20084 15264254

[B45] PiaoL.ChenZ.LiQ.LiuR.SongW.KongR. (2019). Molecular dynamics simulations of wild type and mutants of SAPAP in complexed with Shank3. *Int. J. Mol. Sci.* 20:224. 10.3390/ijms20010224 30626119PMC6337207

[B46] RoskoskiR.Jr. (2013). Anaplastic lymphoma kinase (ALK): Structure, oncogenic activation, and pharmacological inhibition. *Pharmacol. Res.* 68 68–94. 10.1016/j.phrs.2012.11.007 23201355

[B47] Sebastián-SerranoÁDiego-GarcíaD.Díaz-HernándezM. (2018). The neurotoxic role of extracellular tau protein. *Int. J. Mol. Sci.* 19:998. 10.3390/ijms19040998 29584657PMC5979432

[B48] ShivakumarD.WilliamsJ.WuY.DammW.ShelleyJ.ShermanW. (2010). Prediction of absolute solvation free energies using molecular dynamics free energy perturbation and the OPLS force field. *J. Chem. Theory Comp.* 6 1509–1519. 10.1021/ct900587b 26615687

[B49] SinhaS.AndersonJ. P.BarbourR.BasiG. S.CaccavelloR.DavisD. (1999). Purification and cloning of amyloid precursor protein β-secretase from human brain. *Nature* 402 537–540. 10.1038/990114 10591214

[B50] ToscoP.BalleT.ShiriF. (2011). Open3DALIGN: An open-source software aimed at unsupervised ligand alignment. *J. Comp. Aided Mol. Design* 25 777–783. 10.1007/s10822-011-9462-9 21792629

[B51] ToukmajiA. Y.BoardJ. A.Jr. (1996). Ewald summation techniques in perspective: A survey. *Comp. Phys. Commun.* 95 73–92. 10.1016/0010-4655(96)00016-1

[B52] TresadernG.DelgadoF.DelgadoO.GijsenH.MacdonaldG. J.MoecharsD. (2011). Rational design and synthesis of aminopiperazinones as β-secretase (BACE) inhibitors. *Bioorgan. Med. Chem. Lett.* 21 7255–7260. 10.1016/j.bmcl.2011.10.050 22071305

[B53] TrottO.OlsonA. J. (2010). AutoDock Vina: Improving the speed and accuracy of docking with a new scoring function, efficient optimization, and multithreading. *J. Comput. Chem*. 31, 455–461. 10.1002/jcc.21334 19499576PMC3041641

[B54] VassarR.BennettB. D.Babu-KhanS.KahnS.MendiazE. A.DenisP. (1999). β-Secretase cleavage of Alzheimer’s amyloid precursor protein by the transmembrane aspartic protease BACE. *Science* 286 735–741. 10.1126/science.286.5440.735 10531052

[B55] VolkamerA.KuhnD.GrombacherT.RippmannF.RareyM. (2012). Combining global and local measures for structure-based druggability predictions. *J. Chem. Inf. Model* 52 360–372. 10.1021/ci200454v 22148551

[B56] YanR.BienkowskiM. J.ShuckM. E.MiaoH.ToryM. C.PauleyA. M. (1999). Membrane-anchored aspartyl protease with Alzheimer’s disease β-secretase activity. *Nature* 402 533–537. 10.1038/990107 10591213

[B57] YangL. B.LindholmK.YanR.CitronM.XiaW.YangX. L. (2003). Elevated β-secretase expression and enzymatic activity detected in sporadic Alzheimer disease. *Nat. Med.* 9 3–4. 10.1038/nm0103-3 12514700

[B58] ZacchettiD.ChieregattiE.BettegazziB.MihailovichM.SousaV. L.GrohovazF. (2007). BACE1 expression and activity: Relevance in Alzheimer’s disease. *Neurodegener. Dis.* 4 117–126. 10.1159/000101836 17596706

[B59] ZakiM. E. A.Al-HussainS. A.MasandV. H.AkasapuS.BajajS. O.El-SayedN. N. E. (2021). Identification of Anti-SARS-CoV-2 Compounds from Food Using QSAR-Based Virtual Screening, Molecular Docking, and Molecular Dynamics Simulation Analysis. *Pharmaceuticals* 14:357. 10.3390/ph14040357 33924395PMC8070011

[B60] ZhangY. W.ThompsonR.ZhangH.XuH. (2011). APP processing in Alzheimer’s disease. *Mol. Brain* 4:3. 10.1186/1756-6606-4-3 21214928PMC3022812

